RETRACTED

# Shwachman-Diamond Syndrome in a Child Presenting With Chronic Diarrhea: A Rare Case in Family Medicine Practice

**DOI:** 10.7759/cureus.19391

**Published:** 2021-11-09

**Authors:** Malak Alshammari, Malak A Aljohani, Joud M Hashash, Hatim A Alsaedi, Waad Y Alobaidi, Nouf K Alhuzali, Mohammed S Alnumani, Asrar H Alrashidi, Sulaiman A Al-Battniji, Naif A Alotaibi, Nouran K Alhumaidi, Ahmed N Alajaimi, Rawabi S Alqurashi, Abdulrahman T Albishri, Khalid H Alshammari

**Affiliations:** 1 College of Medicine, Imam Abdulrahman Bin Faisal University, Dammam, SAU; 2 College of Medicine, Batterjee Medical College, Jeddah, SAU; 3 College of Medicine, King Saud bin Abdulaziz University For Health Sciences, Riyadh, SAU; 4 College of Medicine, King Saud University, Riyadh, SAU; 5 College of Medicine, King Abdulaziz University, Jeddah, SAU; 6 College of Medicine, Arabian Gulf University, Manama, BHR; 7 College of Medicine, Princess Nourah Bint Abdul Rahman University, Riyadh, SAU; 8 General Practice, King Faisal Military Hospital, Asir, SAU; 9 College of Medicine, Shaqra University, Shaqraa, SAU

**Keywords:** case report, failure to thrive, pancreatic exocrine insufficiency, steatorrhea, chronic diarrhea, shwachman-diamond syndrome

## Abstract

Diarrhea remains an important cause of morbidity and mortality worldwide. Chronic diarrhea often represents a diagnostic challenge for family medicine and pediatric physicians because of its broad spectrum of possible etiologies. The differential diagnoses can be narrowed by taking a detailed history and performing an appropriate physical examination. In general, chronic diarrhea can be due to osmotic, secretory, inflammatory, or dysmotility-related pathologies. We present the case of a 30-month-old male who was brought to the family medicine clinic with a complaint of abdominal bloating and persistent diarrhea after every feeding for four months. His stools were foul-smelling and occurred more than four times a day. The patient was below the second standard deviations for weight and height. He appeared pale, and there was no scleral icterus. The patient underwent upper endoscopy, which showed no abnormal gross findings. A dedicated abdominal computed tomography scan was performed to evaluate the pancreas for any structural abnormalities. The scan demonstrated complete replacement of the pancreatic parenchyma by fatty tissue. The diagnosis of Shwachman-Diamond syndrome was established as the analysis revealed a mutation in the SBDS gene. The patient was treated with pancreatic enzyme replacement therapy. After two months of follow-up, the parents reported that the patient had significant improvement in diarrhea. Shwachman-Diamond syndrome is a very rare inherited disorder characterized by bone marrow failure, exocrine pancreatic dysfunction, and skeletal abnormalities. Despite its rarity, clinicians should keep a high index for this condition when they encounter a child with unexplained chronic diarrhea.

RETRACTED

## Introduction

Diarrhea remains an important cause of morbidity and mortality worldwide. It is estimated that diarrheal illnesses are responsible for approximately four million deaths in children globally [1]. It is the leading cause of mortality among children aged below five years [2]. Diarrhea lasting for more than four weeks is termed chronic diarrhea [3]. Chronic diarrhea often represents a diagnostic challenge for family medicine and pediatric physicians because of its broad spectrum of possible etiologies. The differential diagnoses can be narrowed by taking a detailed history and performing an appropriate physical examination. The appropriate management should be performed with no delays for chronic diarrhea with abnormal growth measurements. The management of diarrhea varies according to the underlying etiology. In general, chronic diarrhea can be due to osmotic, secretory, inflammatory, or dysmotility-related pathologies. Steatorrhea, an abnormal increase in the fat content of the stools, is often related to exocrine pancreatic insufficiency [4]. Here, we present the case of a young child with chronic steatorrhea and abnormal hematological parameters. After a thorough investigation, the patient was diagnosed with Shwachman-Diamond syndrome, a rare inherited disorder.

## Case presentation

We present the case of a 30-month-old male who was brought to the family medicine clinic with a complaint of abdominal bloating and persistent diarrhea after every feeding for four months. His stools were foul-smelling and occurred more than four times a day. The diarrhea was associated with a failure to gain weight. The parents reported that the child has a normal appetite with no history of vomiting or feeding intolerance. There was no history of fever, night sweats, rash, cough, or joint pain. The child did not have any recent sick contact. The patient was seen by several general practitioners for the same complaint, but no diagnosis was obtained.

The patient had an unremarkable past medical history. He did not have any previous hospital admissions. He had no history of previous surgeries. He does not take any medications and was not known to have any food or drug allergies. Regarding the perinatal history, the child was full term with a birth weight of 3.5 kg. The labor and delivery were unremarkable for any complications. The child was up to date with his vaccination schedule. Regarding the developmental history, the child reached the developmental milestones at the appropriate ages, and there was no parental concern regarding his development. The social history was noncontributory. There was no history of diseases running in the family. The child was not born of a consanguineous marriage.

RETRACTED

Upon examination, the child was awake and alert and did not appear sick. No dysmorphic features were noted. The patient was below the second standard deviations for weight and height. He appeared pale, and there was no scleral icterus. His vital signs were as follows: heart rate of 90 bpm, blood pressure of 80/52 mmHg, respiratory rate of 22 bpm, and temperature of 36.8°C. Abdominal examination revealed a soft and non-tender abdomen with no organomegaly and had normal bowel sounds. Neurological examination, including hearing and vision tests, was normal. No evidence of muscle wasting was noted. The cardiorespiratory examination was unremarkable. The initial laboratory investigation revealed a hemoglobin level of 14.1 g/dL, leukocyte count of 5100/µL, and platelet count of 370,000/µL. Liver enzymes were mildly elevated. The total protein was 2.9 g/dL. His random glucose level was normal. Stool analysis, including routine culture, ova, and parasite testing, was negative. Stool testing for reducing substances yielded negative results. The remainder of the laboratory evaluations is summarized in Table 1.

**Table 1:** Summary of the results of the laboratory findings

Laboratory Investigation	Unit	Result	Reference Range
Hemoglobin	g/dL	14.1	13–18
White Blood Cell	1000/mL	5.1	4–11
Platelet	1000/mL	370	140–450
Erythrocyte Sedimentation Rate	mm/hour	5	0–20
C-Reactive Protein	mg/dL	0.4	0.3–10
Total Bilirubin	mg/dL	0.4	0.2–1.2
Albumin	g/dL	2.9	3.4–5
Alkaline Phosphatase	U/L	120	46–116
Gamma-Glutamyl Transferase	U/L	86	15–85
Alanine Transferase	U/L	70	14–63
Aspartate Transferase	U/L	42	15–37
Blood Urea Nitrogen	mg/dL	9	7–18
Creatinine	mg/dL	0.7	0.7–1.3
Sodium	mEq/L	138	136–145
Potassium	mEq/L	3.5	3.5–5.1
Chloride	mEq/L	104	98–107
Anti-endomysial IgA Antibody		Negative	Negative
Antireticulin IgA Antibody		Negative	Negative
Antigliadin IgA		Negative	Negative
Anti-tissue Transglutaminase Antibodies		Negative	Negative

Because of the clinical and laboratory findings, the patient was referred to the pediatric gastroenterology center for further investigation. The patient underwent upper endoscopy, which showed no abnormal gross findings. However, mild duodenal inflammation was evident in the histopathological examination of the obtained specimen. The patient underwent a 72-hour fecal fat collection, which indicated the presence of fat malabsorption. Subsequently, the fecal pancreatic elastase level was measured as 20 fecal μg/g. Such findings were consistent with exocrine pancreatic dysfunction. To exclude the possibility of cystic fibrosis as the underlying etiology of malabsorption, a chloride sweat test was performed and yielded negative results.

RETRACTED

A dedicated abdominal computed tomography scan to evaluate the pancreas for any structural abnormalities was performed. The scan demonstrated complete replacement of the pancreatic parenchyma by fatty tissue (Figure 1). The suggested differential diagnoses by the radiologist for the fatty replacement of the pancreas included cystic fibrosis, Shwachman-Diamond syndrome, and Johanson-Blizzard syndrome. The blood sample of the patient was sent for genetic analysis. The diagnosis of Shwachman-Diamond syndrome was established as the analysis revealed a mutation in the SBDS gene (Table 2). The detected mutation was previously reported in the literature [5].

**Figure 1:** Axial computed tomography image Selected computed tomography axial image of the abdomen with intravenous contrast in the port venous phase demonstrating complete fatty replacement of the pancreatic parenchyma (arrows).

**Table 2:** Information about the genetic analysis results Note: DNAJC21, EFL1, and SRP54 genes were not found to have any pathogenic mutations.

Gene	SBDS Allele 1	SBDS Allele 2
Chromosomal	Chromosome 7	Chromosome 7
Mutation	258+2 T → C	183-184 TA → CT
Site of Mutation	Exon 2	Exon 2
Type of Mutation	Non-sense	Non-sense
Description of Mutation	Deletion of 8 base pairs	Dinucleotide change

The patient was treated with pancreatic enzyme replacement therapy. After two months of follow-up, the parents reported that the patient had significant improvement in diarrhea. A weight gain was observed. Since the patient did not have any history of bleeding or recurrent infections, treatment with granulocyte colony-stimulating factor was not offered.

## Discussion

We presented the case of a 30-month-old male with Shwachman-Diamond syndrome presenting with chronic diarrhea and failure to gain weight. Shwachman-Diamond syndrome is a rare inherited disorder with an incidence of 1 per 150,000 live births [6]. The syndrome is characterized by bone marrow failure, exocrine pancreatic dysfunction, and skeletal abnormalities.

The typical presentation of Shwachman-Diamond syndrome is during early childhood or infancy. It presents with recurrent infections, growth retardation, and failure to thrive. The neutropenia can be intermittent or persistent. The affected patients are at higher risk of infection either because of quantitative or qualitative defects in neutrophils. Most frequent infections include pneumonia, recurrent otitis media, and skin infections [7]. In subsets of patients, the neutropenia may be associated with a varying degree of anemia and thrombocytopenia. According to clinical data from a large international cohort, Ginzberg et al. [5] reported that neutropenia is present in 98%, anemia in 42%, and thrombocytopenia in 34% of patients. In the present case, however, the patient did not exhibit neutropenia on his presentation, and there was no history of recurrent infections.

RETRACTED

Exocrine pancreatic dysfunction is a common presentation of Shwachman-Diamond syndrome, and it was the only manifestation of the syndrome in the present case [5]. The clinical manifestation of pancreatic dysfunction varies significantly in severity. It ranges from the asymptomatic nature to severe dysfunction causing steatorrhea and failure to thrive [8]. It is interesting to note that pancreatic dysfunction may show progressive improvement with age. In the present case, pancreatic imaging guided us to reach the diagnosis. Pancreatic imaging demonstrates a small and shrunken pancreas with lipomatosis or fatty replacement [9].

Different forms of skeletal abnormalities have been described in patients with Shwachman-Diamond syndrome. Such abnormalities include short status, thoracic dystrophies, short arms and legs, and metaphyseal dysplasia. These abnormalities are typically symmetrical. It seems that these abnormalities develop independent of the exocrine pancreatic sufficiency.

The differential diagnoses of Shwachman-Diamond syndrome include other conditions and hematologic, pancreatic, and linear growth disorders. In our case, the patient presented solely with exocrine pancreatic dysfunction. Cystic fibrosis is the most common cause of exocrine pancreatic dysfunction. However, patients with cystic fibrosis present with pulmonary disease and have abnormal sweat chloride tests. Further, Pearson syndrome may be associated with exocrine pancreatic insufficiency, bone marrow failure, and failure to thrive [10]. However, patients with Pearson syndrome tend to have pancreatic fibrosis rather than lipomatosis on pancreatic imaging. Johanson-Blizzard syndrome is an inherited disorder that should be considered as a differential diagnosis of Shwachman-Diamond syndrome. Johanson-Blizzard syndrome, however, is associated with thyroid hormone disturbances, scalp defects, urogenital malformations, and imperforate anus [11]. In addition, several other inherited disorders should be considered in the differential diagnosis of Shwachman-Diamond syndrome depending on the predominantly involved organs.

## Conclusions

Shwachman-Diamond syndrome is a very rare inherited disorder characterized by bone marrow failure, exocrine pancreatic dysfunction, and skeletal abnormalities. Despite its rarity, clinicians should keep a high index for this condition when they encounter a child with unexplained chronic diarrhea. The classic triad of Shwachman-Diamond syndrome may not be present in all patients, and the condition may present with pancreatic dysfunction only. Pancreatic enzyme replacement is the treatment of choice in such cases. As in the present case, imaging for the pancreas by ultrasound, computed tomography, or magnetic resonance imaging can be helpful to suggest the diagnosis.
